# Genetic regulation of murine pituitary development

**DOI:** 10.1530/JME-14-0237

**Published:** 2015-04

**Authors:** Karine Rizzoti

**Affiliations:** Division of Stem Cell Biology and Developmental Genetics, MRC National Institute for Medical Research, The Ridgeway, Mill Hill, London, NW7 1AA, UK

**Keywords:** pituitary, developmental factors, morphogenesis, stem cell

## Abstract

Significant progress has been made recently in unravelling the embryonic events leading to pituitary morphogenesis, both *in vivo* and *in vitro*. This includes dissection of the molecular mechanisms controlling patterning of the ventral diencephalon that regulate formation of the pituitary anlagen or Rathke's pouch. There is also a better characterisation of processes that underlie maintenance of pituitary progenitors, specification of endocrine lineages and the three-dimensional organisation of newly differentiated endocrine cells. Furthermore, a population of adult pituitary stem cells (SCs), originating from embryonic progenitors, have been described and shown to have not only regenerative potential, but also the capacity to induce tumour formation. Finally, the successful recapitulation *in vitro* of embryonic events leading to generation of endocrine cells from embryonic SCs, and their subsequent transplantation, represents exciting advances towards the use of regenerative medicine to treat endocrine deficits. In this review, an up-to-date description of pituitary morphogenesis will be provided and discussed with particular reference to pituitary SC studies.

## Introduction

The pituitary is a small endocrine gland encased in a depression of the sphenoid bone called the sella turcica, at the base of the skull, just under a part of the brain called the hypothalamus to which it is physically linked by the pituitary stalk. This connection between the pituitary and the hypothalamus is crucial, initially in the embryo for correct morphogenesis of both components of the hypothalamo–pituitary axis, and also postnatally because the hypothalamus controls the secretions of the gland through this stalk. In the embryo, development of the pituitary anlagen or Rathke's pouch (RP) depends on the inductive actions of a restricted domain of the developing ventral diencephalon (VD) with which it is in contact, the infundibulum. It will give rise to the pituitary stalk and neurohypophysis (posterior pituitary). After birth, the different nuclei or groups of neurons that constitute the hypothalamus sense peripheral information, directly and/or indirectly via other parts of the brain, and accordingly secrete specific neurohormones (Fig. 1).

One important function of the hypothalamo–pituitary axis is to maintain a general internal equilibrium or homoeostasis. However, it also ensures that the organism responds appropriately to changing physiological situations such as puberty, pregnancy, lactation, and also to stress. An important feature of the system is therefore its plasticity with hormonal secretions being constantly modulated. The seven different hormones secreted by the pituitary affect most physiological processes. It is therefore not surprising that pathological situations leading to pituitary hormone imbalance have pleiotropic consequences resulting in significant morbidity and even mortality. Hormone deficiencies (those affecting more than one hormones are described as combined pituitary hormone deficiencies (CPHD)) can be congenital or acquired, and these can have a pituitary or hypothalamic origin and are, in most cases, of unknown aetiology (Kelberman *et al*. 2009). The most frequent congenital defect in humans is isolated growth hormone (GH) deficiency with a prevalence of one in 3500–10 000 births (Kelberman *et al*. 2009). Acquired deficits develop mainly as a consequence of pituitary tumours (mostly prolactinomas) and brain damage (Hannon *et al*. 2013). Substitution or replacement therapies are available to treat deficiencies but these are not optimal because they do not reproduce the physiological secretion patterns, are associated with side effects, and are costly.

Stem cells (SCs) are present in most tissues and organs and are characterised by their capacity to both self-renew and give rise to differentiated progeny, according to the tissue/organ they belong to. Such cells have been recently characterised in the pituitary (Andoniadou *et al*. 2013, Rizzoti *et al*. 2013). In organs with a rapid turnover such as the intestine and the haematopoietic system, they are required for tissue homoeostasis and are also recruited in response to physiological challenges, such as injuries. In organs with a low turnover such as the brain and the pituitary (Levy 2002), they can provide a source of differentiating cells to replace those lost through normal processes of attrition, but they mostly appear to be mobilised in response to physiological challenges or to damage (Fu *et al*. 2012, Langlais *et al*. 2013, Rizzoti *et al*. 2013). SCs can also be involved in tumourigenesis, when self-renewal becomes abnormal. In some cases, they can transform into cancer SCs that provide tumours with a pool of reserve cells that can sustain their growth by differentiating into ‘bulk’ tumour cells, and also allow their recurrence after therapy (for review, see Kreso & Dick (2014)). In other cases, SCs can induce formation of tumours in neighbouring cells, and this has been shown in particular in the pituitary (Andoniadou *et al*. 2013).

Regenerative medicine based on SC therapies holds promise for many diseases and injuries, where lost functions could be restored by supplying SCs or their differentiated derivatives. In the pituitary, the ability to replace missing endocrine cells would represent a significant improvement to treat long-term pituitary deficiencies. Developmental mechanisms are often, but not always (Lepper *et al*. 2009), re-capitulated in adult SCs for self-renewal, differentiation and also during oncogenic transformation. In this review, an up-to-date description of pituitary morphogenesis will be provided, highlighting the latest developments. Finally, recent pituitary SC studies and advances towards regenerative therapies will be discussed.

## Pituitary morphology and morphogenesis

### Morphology

The pituitary gland is composed of three different lobes: anterior, intermediate and posterior (Fig. 1). The anterior lobe is the largest and it is richly vascularised by capillaries that deliver hypothalamic inputs and send secreted hormones from five different populations of endocrine cells (Fig. 1). It has been recently demonstrated that endocrine populations form homotypic networks ensuring a robust and coordinated hormonal secretory response to stimulation (for review, see Mollard *et al*. (2012)). These networks are plastic and can be modulated according to physiological contexts (Hodson *et al*. 2012). Pituitary SCs/progenitors are localised around the pituitary cleft, a remnant of the RP lumen, and scattered in the anterior lobe (for review, see Rizzoti (2010), Castinetti *et al*. (2011*a*) and Vankelecom (2012)). They at least partially overlap with folliculo-stellate cells, a heterogeneous population of dendritic cells (Fauquier *et al*. 2008, Andoniadou *et al*. 2013). Pituitary SCs also appear to form a network but its functionality has not yet been studied (Mollard *et al*. 2012).

The intermediate lobe is located between the anterior and the posterior lobes. It contains only one endocrine population, the melanotrophs. This lobe is poorly vascularised and receives hypothalamic information by direct hypothalamic innervation. Capillaries located between IL and PL collect hormones. It is a useful model for cancer formation in rodents as mutants for several cell cycle regulators display intermediate lobe tumours (for review, see Quereda & Malumbres (2009)). In humans, this lobe is only residual and melanotrophs are mainly found in the skin.

The posterior lobe does not contain any endocrine cells but a population of glial cells called pituicytes and axonal termini from two types of hypothalamic neurons.

Despite being closely associated, the three pituitary lobes do not have the same embryonic origin. Anterior and intermediate lobes, forming the anterior pituitary, are ectodermal derivatives while the posterior lobe has a neuroectodermal origin.

### Morphogenesis

Cells secreting peptides related to pituitary hormones exist in invertebrates but the gland is specific to vertebrates (for review, see Patthey *et al*. (2014)). Pituitary development is initiated during neurulation, from 8 days post coitum (dpc) in mice (all stages refer to mouse development). An ectodermal thickening or hypophyseal placode (HP) appears in the rostral most position, within the anterior neural ridge, which forms just in front of the future VD (Fig. 1). HP forms along with other sensory placodes (olfactory, optic and otic) and it has been proposed that olfactory and HPs were fused into one nasoHP in ancestral craniates. Separation and the subsequent duplication of the olfactory placodes on each side of the median HP have been suggested to represent an important event during evolution, because it allowed development of the future jaws (Khonsari *et al*. 2013).

By 9 dpc, the future telencephalon has grown relatively faster than the diencephalon and fused rostrally at the midline, so that the future brain is now bent at the level of the diencephalon. As a consequence, the diencephalon is shifted posteriorly. HP has morphed into the pituitary anlagen or RP, an epithelial invagination that forms in continuity with the oral ectoderm and extends dorsally towards VD. RP is located at an interesting junction. It marks the posterior limit of neural crest cell (NCC) contribution to the head mesenchyme; therefore, it is flanked anteriorly by NCC-derived mesenchyme and posteriorly by mesoderm-derived mesenchyme (Jiang *et al*. 2002). It is in contact with the anterior border of foregut endoderm (Khonsari *et al*. 2013), and it is also located just in front of the notochord and importantly it is directly in contact with VD. RP is therefore exposed to signals secreted from all the different territories it is in contact with, and these are important for proper morphogenesis.

By 10 dpc, the region of VD directly above RP starts to evaginate towards it. This territory is the infundibulum, which will give rise to the median eminence, pituitary stalk and posterior lobe (for review, see Pearson & Placzek (2013)), while RP will form the anterior and intermediate lobes. The connection between RP and oral ectoderm disappears through apoptosis (Charles *et al*. 2005). In ancestral vertebrates, this link was maintained as the buccohypophyseal canal, which may have been involved in osmoregulation in some species (Khonsari *et al*. 2013).

The mature pouch is initially formed of highly proliferative epithelial progenitors arranged around the lumen. Birth dating studies have revealed that there is a main wave of mitotic exit between 11.5 and 13.5 dpc regardless of the endocrine cell type (Davis *et al*. 2011), while differentiation, characterised by expression of the secreted hormone, occurs at a different time for each population (Japon *et al*. 1994). Undifferentiated cells exiting the cell cycle adopt more ventral and lateral locations and lose epithelial characteristics, reminiscent of epithelial-to-mesenchymal transition (Himes & Raetzman 2009). All endocrine cell types are present before birth, but cells fully differentiate only postnatally as the secretory apparatus further matures and cell size increases. Homotypic endocrine networks form in the embryo, starting with corticotrophs, where single cells initially arrange into clusters shortly after differentiation. These may serve as a scaffold for the organisation of other endocrine populations (Budry *et al*. 2011*a*).

In rodents, the gland will undergo a phase of important growth during the 1st weeks of life. This is characterised by high levels of proliferation, both in progenitors and in endocrine cells. Throughout life, endocrine cells retain the capability to proliferate but they do so very rarely (Levy 2002). After birth, the hypothalamus will take control of pituitary endocrine maturation and secretions, but it is not clear exactly when and how its influence starts to be exerted.

## Genetic regulation of pituitary development

### Induction of the pituitary primordium, the HP

Just after gastrulation, complex interactions between the head mesoderm and the neural and non-neural ectoderm define a domain at the border of the neural plate. These involve fibroblast growth factor (FGF) signalling inducing neural fate, bone morphogenetic proteins (BMPs) and wingless-related integration site (WNT) activities inducing future epidermal identity in non-neural ectoderm, and active inhibition of BMP and WNT signalling pathways by the neural ectoderm and head mesoderm (for review, see Saint-Jeannet & Moody (2014)). Within this domain, cells are competent to become either placodal or NCC. Rostrally, individual placodes are further specified by surrounding tissues.

While the head ectoderm is generally competent to form pituitary tissue, the inducing ability is restricted to VD, which is required for HP induction and maintenance (elAmraoui & Dubois 1993, Kawamura & Kikuyama 1998, Gleiberman *et al*. 1999). Foregut endoderm is also likely to be involved in early pituitary development, either directly because it is in contact with the pituitary primordium (Khonsari *et al*. 2013) or indirectly because it is necessary for anterior neural plate patterning (Thomas & Beddington 1996).

Several transcription factors expressed early in HP are required for later pituitary development. The paired-like homoeodomain transcription factor HESX1 is an important regulator of anterior development (Hermesz *et al*. 1996, Thomas & Beddington 1996, Dattani *et al*. 1998). The Sine Oculis homoeodomain proteins SIX3 and SIX6 (Oliver *et al*. 1995, Jean *et al*. 1999) are also present in the pan-placodal domain and subsequently in the HP (for review, see Schlosser *et al*. (2014)). Finally, but not exhaustively, the homoeodomain transcription factors PITX1 and PITX2 are also present at these early stages (for review, see Soukup *et al*. (2013)).

### Formation and maintenance of RP

#### Signalling pathways

Secreted signals, mainly by VD, are crucial for induction and maintenance of RP (Fig. 2). In addition, several signalling pathways are also active within RP. These will be discussed in this review with an emphasis on recent studies (for review, see Kelberman *et al*. (2009) and Davis *et al*. (2013)).

##### Bone morphogenetic proteins

BMPs are secreted ligands, which upon binding to receptor serine–threonine kinases initiate an intracellular signalling cascade resulting in activation of SMADs and regulation of gene transcription. BMPs are involved in multiple events in the embryo, and dysregulation of the pathway is linked to diseases and cancers (for review, see Cai *et al*. (2012)).

BMP4 is the earliest VD signalling molecule known to be extrinsically required for RP development, from 8.5 dpc (Ericson *et al*. 1998, Takuma *et al*. 1998). It is maintained in the infundibulum with a sharp ventral boundary up to at least 14.5 dpc (Ericson *et al*. 1998, Treier *et al*. 1998, Davis & Camper 2007). In the chick, BMPs are required for infundibular identity and patterning, in particular by inducing expression of the T-box transcription factor TBX2 that represses *Sonic Hedgehog* (*SHH*) expression, excluding it from the future infundibulum (Manning *et al*. 2006). *Bmp2* and *Bmp7* are first present in ventral mesenchyme at 10.5 dpc, then *Bmp2* starts to be expressed in RP, first ventrally and then throughout, decreasing by 14.5 dpc (Ericson *et al*. 1998, Davis & Camper 2007). The pattern of phosphorylated SMADs between 10.5 and 14.5 dpc correlates with the presence of BMP2 (Davis *et al*. 2011). Conditional deletion of the gene encoding its receptor, *Bmpr1a*, in RP at 9.5 dpc results in underdevelopment of the pouch at 10.5 dpc. Therefore, BMP signalling is intrinsically required for RP maintenance and probably for progenitor proliferation (Davis & Camper 2007).

##### Fibroblast growth factors

FGFs are secreted molecules that bind to receptor tyrosine kinases resulting in activation of multiple signalling cascades through MAPK, PI3 kinase and phospholipase C, affecting, respectively, cell proliferation, survival and motility (for review, see Dorey & Amaya (2010)). They are required for multiple processes during embryogenesis, and dysregulation is linked to cancer and many congenital diseases such as Kallmann syndrome, which affects differentiation of gonadotrophin-releasing hormone (GnRH) neurons (GnRH is a hypothalamic neuropeptide required for reproductive development and function) resulting in hypogonadism (for review, see Chung & Tsai (2010)).

During RP development, *Fgf8*, *Fgf10* and *Fgf18* are present in VD, appearing later than *Bmp4*, from 9.5 dpc up until at least 14.5 dpc (Ericson *et al*. 1998, Treier *et al*. 1998, 2001). In chick, FGFs are required within the infundibulum for cell expansion (Pearson *et al*. 2011). In the murine RP, MAPK activation is observed dorsally between 10.5 and 11.5 dpc in agreement with an infundibular source of FGFs (Davis *et al*. 2011). Deletion of *Fgf10* or *Fgfr2IIIb* results in formation of a small apoptotic pouch (De Moerlooze *et al*. 2000, Ohuchi *et al*. 2000). In contrast, deletion of the paired homoeodomain transcription factor *Vax1*, normally expressed in VD but excluded from the infundibulum, causes the appearance of a second *Fgf10*-expressing, but *Bmp4*-negative, anterior domain, disconnected from the infundibulum. This results in induction of a second RP, leading to duplication of the pituitary (Bharti *et al*. 2011). FGFs are therefore necessary for dorsal RP progenitor proliferation and maintenance. By analogy to other models, where FGFs act as chemoattractants (for review, see Friedl & Gilmour (2009)), they may also be involved in RP invagination.

##### Sonic hedgehog

Hedgehog (HH) ligands (Sonic, Desert and Indian hedgehog) not only have been described as morphogens in the embryo, but also act as mitogens, in particular for adult SCs. In the absence of ligand, the receptor Patched inhibits the transmembrane molecule smoothened (SMO), and intracellular GLI repressors silence target genes. In the presence of Hh, SMO allows Gli activators to translocate to the nucleus and activate target gene expression. Dysregulation of SHH signalling results in holoprosencephaly, a syndrome characterised by severe midline defects (Chiang *et al*. 1996). Postnatally, dysregulation of the pathway is linked to several cancers (for review, see Athar *et al*. (2014)).

Within the ventro-medial diencephalon, SHH is present anteriorly and laterally to the infundibulum, from which it is excluded (Manning *et al*. 2006, Trowe *et al*. 2013). Within the antero-ventral domain, it is required for maintenance of the prospective hypothalamus. Its expression in this domain depends on the HMG box transcription factors *Sox2* and *Sox3* (Zhao *et al*. 2012). Exclusion of SHH from the infundibulum is achieved by sequestration of SOX2/SOX3 away from a *Shh* enhancer by TBX2/TBX3 (Trowe *et al*. 2013). In the absence of SHH in VD, infundibular *Bmp4* and *Fgf10* patterns are expanded ventrally, resulting in an anterior shift and duplication of RP. In contrast, when *Tbx3* is deleted, the *Shh* domain is expanded dorsally. *Fgf8* and *Bmp4* are still expressed while *Fgf10* is down-regulated in the infundibulum, where more proliferation is observed. Moreover, evagination fails and consequently RP does not progress beyond 10.5 dpc (Trowe *et al*. 2013). Altogether, these studies suggest an antagonism between BMP and SHH in VD that is required for infundibular morphogenesis and hence RP positioning and development (Zhao *et al*. 2012, Trowe *et al*. 2013).

SHH is also present in the oral ectoderm, but excluded from RP (Treier *et al*. 2001). It has recently been proposed that SHH is involved in individualisation of RP from the oral ectoderm as dysregulation of the SHH pathway in human and mouse results in maintenance of an ancestral link between RP and oral ectoderm, the buccohypophyseal canal. In consequence, the pituitary in such mutants is ventrally displaced just above the oral cavity and sometimes even connected to it (Khonsari *et al*. 2013). SHH is therefore likely to be required in the oral ectoderm for basal skull and pituitary morphogenesis.

Within RP, cells express the receptor Patched and the transcriptional regulators GLI1, GLI2 and GLI3; therefore, they are competent to respond to the ligand (Treier *et al*. 2001). Conditional deletion of *Gli2* and *Gli3* in RP has revealed that the pathway is involved in RP progenitor proliferation (Wang *et al*. 2010).

In conclusion, the SHH pathway has different roles, being required in VD, in oral ectoderm and finally within RP for proper pituitary morphogenesis.

##### WNT

The WNT-secreted molecules play important roles in the embryo and in the adult, regulating in particular proliferation of different SC populations. Dysregulation of the pathway is causative of many diseases, especially colorectal cancers (for review, see Clevers & Nusse (2012)). The canonical WNT pathway is characterised by the central role of the intracellular protein β-catenin. In the absence of the ligand, β-catenin is targeted for degradation. When WNT binds to the co-receptors LRP5/LRP6 and receptor Frizzled, cytoplasmic β-catenin can accumulate and translocate to the nucleus where it displaces the repressor Groucho, associated with the T-cell factor/lymphoid enhancer-binding factor (TCF/LEF) transcription factors. WNT target genes that were silenced can now be activated. A second WNT-activated pathway regulates planar cell polarity, affecting cell morphology and movement, and a third is the related non-canonical Wnt pathway, associated with intracellular Ca^2+^ release.

WNT5a, along with other members of the pathway, is present throughout VD and RP from 9.5 to 12.5 dpc (Treier *et al*. 1998, Cha *et al*. 2004, Potok *et al*. 2008). In its absence, the β-catenin activation pattern is unaffected, suggesting that Wnt5a does not activate the canonical pathway, but infundibular signalling is ectopically expanded ventrally (Potok *et al*. 2008). This results in more oral ectoderm being recruited to form RP and with the appearance of extrabifurcations (Cha *et al*. 2004). Cell fate is unaffected in RP; therefore, WNT5A may be necessary in VD for correct patterning and indirectly affects RP shaping (Potok *et al*. 2008). TCF4 is also expressed in VD and RP. Deletion of the gene results in a similar phenotype as *Wnt5a* ablation, but deletion of TCF/LEF factors is not necessarily comparable to loss of ligand or of β-catenin, because these actively repress transcription when the pathway is inactive. Both proteins are probably independently involved within VD in patterning and hence RP positioning.

Within RP, several WNT ligands and members of the pathways are present and active (Olson *et al*. 2006, Potok *et al*. 2008). Deletion of *Wnt4*, which is usually expressed transiently and exclusively in RP, causes a slight reduction in expression of the transcription factor PIT required for emergence of somatotrophs, lactotrophs and thyrotrophs (Potok *et al*. 2008). Derepression of target genes in *Tcf4*-deleted mutants may underlie the observed over-proliferation phenotype in the pouch. In these mutants, endocrine cell differentiation can still occur (Brinkmeier *et al*. 2007). There is, however, little nuclear β-catenin staining in RP (Brinkmeier *et al*. 2007), and deletion of the gene encoding this does not, at least initially, cause any defect (Olson *et al*. 2006). β-catenin has nonetheless been demonstrated to participate in *Pitx2* activation (Kioussi *et al*. 2002, Ai *et al*. 2007), which in turn stimulates progenitor proliferation, but the identity of the Wnt ligand is unknown (Kioussi *et al*. 2002). Later on, β-catenin can interact with the transcription factor PROP1 (see below) and formation of this complex is important for emergence of endocrine lineages (Olson *et al*. 2006). Moreover, constitutive activation of the pathway, using a β-catenin degradation resistant form under the control of a portion of the *Pitx1* promoter as a transgene, results in loss of the pituitary at 13.5 dpc (Olson *et al*. 2006). In contrast with this last result, two recent studies have demonstrated that conditional expression of a constitutively active β-catenin mutant protein in response to Cre-mediated activation with either *Hesx1*^*Cre*^ or *Sox2*^*CreERT2*^ (both targeted alleles) caused increased proliferation, reduction in GH content, and importantly, development of tumours, similar to human craniopharyngioma (Gaston-Massuet *et al*. 2011, Andoniadou *et al*. 2013). In conclusion, the WNT canonical pathway may participate in progenitor proliferation and fate while dysregulation of the pathway is clearly linked to oncogenicity.

##### NOTCH

The NOTCH signalling pathway has classically been described in the context of lateral inhibition, where cells within a population are selected to adopt certain alternate fates. Briefly, the membrane-bound ligands Delta-like or Jagged activate the transmembrane receptor NOTCH on neighbouring cells; imbalance between secretion of the ligand and activation of the receptor underlines the cell selection process. Binding of the ligand allows for cleavage of the NOTCH intracellular domain (NICD) that can then translocate to the nucleus, where it displaces repressors such as N-COR that are otherwise associated with the transcription factor RBPJκ when the pathway is inactive. This in turn permits transcriptional activation of targets such as the HES bHLH transcription factors. The pathway is required in the embryo in different contexts and dysregulation is associated not only with inherited and degenerative diseases, but also with cancers in humans (for review, see Hori *et al*. (2013)).

The role of the NOTCH signalling pathway in early VD formation is not fully understood, but it is required for infundibular morphogenesis. *Hes1* is expressed throughout the VD and *Hes* null mutants display reduced evagination and later absence of the PL (Zhu *et al*. 2006, Kita *et al*. 2007, Raetzman *et al*. 2007, Aujla *et al*. 2011).

Several members of the NOTCH pathway are expressed in RP, becoming largely restricted to perilumenal progenitors as the gland develops (Raetzman *et al*. 2004, Zhu *et al*. 2006). Studies of their role demonstrate that they are required for progenitor proliferation and cell fate choice, but different experimental strategies (straightforward deletion, conditional deletion and over activation) lead to different outcomes that are not always reconcilable. Deletion of *Hes* genes result in increased apoptosis and reduced proliferation, inducing pituitary hypoplasia, but AL cell types can differentiate (Raetzman *et al*. 2004, 2007, Kita *et al*. 2007, Monahan *et al*. 2009), with corticotrophs appearing precociously (Zhu *et al*. 2006, Kita *et al*. 2007). The intermediate lobe is more affected, because single or double deletions of the genes encoding the HES1 and HES5 repressors result in either its absence (Zhu *et al*. 2006, Kita *et al*. 2007) or, on a different genetic background, in a hypoplastic appearance with ectopic somatotrophs (Raetzman *et al*. 2007). In contrast, deletion of *Rbpj*κ in RP does not affect intermediate lobe formation, but, as with *Hes* gene deletions, it results in premature and increased corticotroph differentiation with overall reduced proliferation (Zhu *et al*. 2006). Moreover, conditional deletion of either *Rbpj*κ or *Notch2* in RP results in down-regulation of the transcription factor PROP1 (Zhu *et al*. 2006, Nantie *et al*. 2014).

The NOTCH pathway is likely to directly activate *Prop1* expression and this is necessary for emergence of the Pit1 lineage (see above), the latter being absent in *Rbpj*κ mutant pituitaries (Zhu *et al*. 2006). Conversely, regulation of *Notch2* by PROP1 has also been suggested (Raetzman *et al*. 2004). In support of an interaction between the PROP1 and NOTCH pathways, disruption of both *Hes1* and *Prop1* results in a new phenotype with premature corticotroph and αGSU-positive cell differentiation (Himes & Raetzman 2009). Ectopic activation of NOTCH signalling can be achieved by inducing expression of the NICD. Transgenic expression of NICD under control of a *Pit1* (*Pou1f1*) (Zhu *et al*. 2006, Goldberg *et al*. 2011) or a *Pomc* (Zhu *et al*. 2006, Goldberg *et al*. 2011) promoter results in blockade of differentiation. Finally, global impairment of endocrine differentiation results in up-regulation of NOTCH pathway components (Wang *et al*. 2007, Welcker *et al*. 2013). Therefore, NOTCH signalling appears to be required early to prevent differentiation, ensuring the generation of sufficient progenitors, and later to promote emergence of the Pit1 lineage (Zhu *et al*. 2006, Himes & Raetzman 2009), although this later role does not require either HES1 or HES5.

#### Transcriptional regulators

Several transcriptional regulators are required within RP for proper development. Among them, some are additionally present in VD, where they are necessary for infundibular morphogenesis and therefore indirectly for RP morphogenesis. Finally, others are exclusively present and required in VD and affect indirectly the developing pituitary. All of these will be reviewed in this section.

##### HESX1

HESX1 is a paired-like homoeodomain transcription factor that acts as a repressor by co-binding TLE1 (a mammalian Groucho family member) and the nuclear co-repressor N-COR (Dasen *et al*. 2001, Carvalho *et al*. 2010). Human *HESX1* mutations are associated with Septo-optic dysplasia, a rare congenital syndrome characterised by variable CNS midline defects and hypopituitarism (Dattani *et al*. 1998). HESX1 is essential for correct development of the forebrain, and *Hesx1* null mice display postnatal lethality probably caused by CNS defects comprising anophthalmia, a reduced prosencephalon and pituitary dysplasia (Dattani *et al*. 1998). Loss of HESX1 in the anterior neuroectoderm results in posteriorisation due to lack of repression of the Wnt/β-catenin pathway (Andoniadou *et al*. 2007, 2011, Matsuda & Kondoh 2014). The development of RP in *Hesx1* null embryos is characterised early on by a variable phenotype comprising multiple clefts, correlating with expanded infundibular *Fgf10* expression, overproliferation and often misplacement of the gland in the naso-pharyngeal cavity, aspects of which are likely to be explained by loss of the gene in VD (Dasen *et al*. 2001). After birth, hypoplasia of the pituitary is observed and this is suggested to result from impaired hypothalamic control (Gaston-Massuet *et al*. 2008).

*Hesx1* is expressed in RP progenitors until 13.5 dpc (Hermesz *et al*. 1996, Thomas & Beddington 1996). Its expression is activated by the Lim homoeodomain transcription factor LHX3, along with PITX2 and GATA2/GATA3 (Chou *et al*. 2006), while it is down-regulated by the β-catenin/PROP1 complex (Olson *et al*. 2006). *Hesx1* mutant analysis indicates that the interaction of the protein with the repressor TLE1 is crucial for RP development, because the HESX1/TLE1 complex represses expression of *Prop1*, which is necessary for pituitary development to progress (see below) (Dasen *et al*. 2001). Conditional deletion of *Hesx1* in the CNS vs pituitary has not been performed yet to clearly separate both functions, but it has been proposed that lack of repression of the Wnt pathway, as has been observed in the anterior neutral plate, underlies the pituitary phenotype. However, while in neural ectoderm, this results in posteriorisation, in RP the consequence is hyper-proliferation, which has been observed in some of the mutants (Gaston-Massuet *et al*. 2008). Despite these defects, endocrine cell differentiation occurs normally in *Hesx1* mutants, but with increased numbers (Dasen *et al*. 2001, Sajedi *et al*. 2008). HESX1 is therefore an important regulator of early pituitary development and its interaction with PROP1 regulates RP development.

##### SIX3/SIX6

SIX proteins are members of the Sine Oculis homoeobox transcription factor family, present from flatworms to humans. They are well known for their conserved function in eye development and have other important roles during embryogenesis. As regulators of proliferation, they are also involved in tumourigenesis. They can positively or negatively regulate transcription, as they can, respectively, interact with the Eye-absent (EYA) transcriptional activators or the GROUCHO/TLE and DACH co-repressors (for review, see Kumar (2009)). The closely related *Six3* and *Six6* are both expressed in VD and RP (Jean *et al*. 1999, Larder *et al*. 2011), and SIX6 expression is maintained in the adult pituitary (Li *et al*. 2002). Deletion of *Six6* results in formation of hypomorphic pituitaries and retinas. It has been suggested that SIX6 promotes proliferation of progenitors by repressing expression of the cell cycle negative regulator p27KIP1, and such an interaction has been demonstrated to underlie the *Six6*^*−/−*^ retinal phenotype (Li *et al*. 2002).

Deletion of *Six3* is more deleterious and mutants arrest before pituitary development is initiated, and later functions of the gene are not known. However, the phenotype of compound double heterozygous *Six3*; *Hesx1* mutants suggests an interaction of SIX3 with Wnt signalling in RP. In the forebrain, defects in *Six3*^*−/−*^ mutants are more severe than those observed in *Hesx1* mutants, but they are similar and both are proposed to stem from ectopic Wnt/βcatenin activation (Lavado *et al*. 2008, Andoniadou *et al*. 2011). Intriguingly, *Six3*^*+/−*^*; Hesx1*^*+/−*^ RP display increased early progenitor proliferation and multiple clefts, comparable to *Hesx1*^*−/−*^ mutants. This hyper-proliferation phenotype is proposed to result from increased Wnt signalling (Gaston-Massuet *et al*. 2008). Therefore, SIX3 would normally serve as a repressor of Wnt activity. Conditional mutation is now required to assess its function directly.

##### PITX1/PITX2

The paired homoeodomain PITX proteins are important morphogenetic regulators for different organs. They are also well known for their role in left–right asymmetry (for review, see Soukup *et al*. (2013)). *PITX2* mutations are associated with Axenfeld–Rieger syndrome, mainly characterised by eye defects and also comprising pituitary abnormalities. PITX1 and PITX2 are present in the HP, RP and later maintained in differentiated endocrine cells (Gage & Camper 1997, Lanctot *et al*. 1997). They function redundantly and are required for maintenance of early RP progenitors (Charles *et al*. 2005). PITX2 appears to be initially more important, because RP development is arrested in *Pitx2*^*−/−*^ mutants, while *Pitx1* null mutants display a normal RP. *Pitx2* has been shown to be a target of Wnt signalling and to induce progenitor proliferation through direct transcriptional activation of cyclins (Kioussi *et al*. 2002, Ai *et al*. 2007). In *Pitx1*; *Pitx2* double mutants, there is increased cell death and LHX3, which is also required for progenitor maintenance (Zhao *et al*. 2006), is completely down-regulated (Charles *et al*. 2005). Other targets of PITX proteins could underlie this phenotype: indeed, during myogenic differentiation, as metabolic status changes, PITX2 and PITX3 regulate mitochondrial function and anti-oxidant enzymes; in their absence, DNA damage accumulate and apoptosis occurs (L'Honore *et al*. 2014). Proper *Pitx* gene dosage is required throughout development for generation and/or maintenance of endocrine cell numbers (Suh *et al*. 2002). PITX1 and PITX2 are also redundantly required postnatally, for thyrotroph function (Castinetti *et al*. 2011*b*). In conclusion, PITX1 and PITX2 are required not only for pituitary morphogenesis but also for endocrine function, reflecting their many interacting partners and, in consequence, target genes.

##### ISLET 1

Insulin gene enhancer protein ISL-1 (ISLET1) is a LIM-homoeodomain transcription factor, essential for cell fate decisions in different embryonic and SC contexts. ISL1 is expressed throughout the oral ectoderm at 8.5 dpc, maintained in RP at 9.5 dpc and finally further ventrally restricted between 10.5 and 11.5 dpc in prospective rostral tip thyrotrophs (Ericson *et al*. 1998). In the adult gland, it is maintained in gonadotrophs (Schang *et al*. 2013). Its expression in RP could be regulated by BMPs (Davis & Camper 2007), where it is proposed to participate in *Lhx3* activation, along with PITX1 (Mullen *et al*. 2012). *Isl1* null embryos die at 10 dpc and display a severely hypoplastic RP, suggesting that the protein is initially required for progenitor maintenance (Takuma *et al*. 1998).

##### LHX2/LHX3/LHX4

LHX2, LHX3 and LHX4 also belong to the LIM-homoeodomain transcription factor family. LHX2 is expressed throughout VD during RP development and required for infundibulum and hence posterior lobe formation (Zhao *et al*. 2010). As observed in *Tbx3* mutants (Trowe *et al*. 2013), in *Lhx2* null mutants the infundibulum fails to evaginate and proliferate more. Additionally, *Bmp* and *Fgf* expression patterns are ventrally expanded. As a consequence, RP fails to expand dorsally and rather develop more rostrally. Importantly, cell differentiation is unaffected and all endocrine cell types are observed (Zhao *et al*. 2010).

LHX3 and LHX4 are required for both CNS and pituitary development. Mutations in human *LHX3* and *LHX4* are associated with CPHD. Both genes are first expressed in RP at 9.5 dpc. *Lhx4* is subsequently restricted to the future AL then down-regulated at 15.5 dpc, while *Lhx3* is maintained throughout in the adult gland (Sheng *et al*. 1997). LHX4 may participate, along with PROP1 in activation of *Lhx3* expression, as *Lhx4*^*−/−*^; *Prop1*^*−/−*^ mutants, and in contrast with single mutants, do not express LHX3 (Raetzman *et al*. 2002). Initially, the two proteins function redundantly, as shown by gene deletion studies (Sheng *et al*. 1997), where increased apoptosis is a major consequence (Raetzman *et al*. 2002, Ellsworth *et al*. 2008). However, while *Lhx4*^*−/−*^ hypoplastic pituitaries contain all endocrine cell types, in *Lhx3*^*−/−*^ mutants, deficiencies in all cell lineages are observed. This reflects the requirement for LHX3 in the activation of several pituitary hormones, hypothalamic peptide receptors and transcription factors (for review, see Prince *et al*. (2011)). Additionally, expression of *Notch2* is absent in *Lhx3* mutants and this could underlie some of the differentiation defects (Ellsworth *et al*. 2008). Therefore, LHX3 and LHX4 are initially required for progenitor maintenance rather than proliferation and later; LHX3 is also required for proper endocrine differentiation.

##### RX/RAX

Retina and anterior neural fold homeobox protein (RX/RAX) is a paired-like homoeodomain protein, mostly known for its conserved function for eye morphogenesis. It is expressed early in the anterior neural plate, and some null mutants lack part of the forebrain. It is also maintained later in VD, and its deletion, in a second class of null mutants, causes abnormal morphogenesis with lack of infundibular evagination and down-regulation of *Fgf10* expression from 10.5 dpc. Consequently, RP fails to develop beyond this stage and remain fused to oral ectoderm (Medina-Martinez *et al*. 2009). It is also important for later hypothalamic morphogenesis (Lu *et al*. 2013).

##### SOX2/SOX3

The HMG box SOXB1 factors SOX2 and SOX3 are broadly expressed in progenitors in the CNS, where they generally, but not exclusively, promote an undifferentiated proliferative state (for review, see Sarkar & Hochedlinger (2011)). SOX2 is also required for pluripotent cell types in the early embryo, and homozygous null mutant mouse embryos die around implantation. In humans, heterozygous *SOX2* loss-of-function mutations are associated with anophthalmia (Fantes *et al*. 2003) and hypogonadotrophic hypogonadism (reduced gonadal function of hypothalamic origin) (Kelberman *et al*. 2006), while both *SOX3* deletions and duplications are linked to mild hypopituitarism (Laumonnier *et al*. 2002). SOX proteins act with co-factors; therefore, the specificity of their action often relies on their partner(s). Moreover, there is redundancy within a sub-family. Nevertheless, the ‘dose’ of SOXB1 is important. This is true in VD, where both SOX2 and SOX3 are expressed, while, in RP, SOX2 is the only SOXB1 member to be present. In VD, they have been shown to activate the same targets: *Shh*, as mentioned earlier (Zhao *et al*. 2012), and also *Six3* and *Six6* (Lee *et al*. 2012, 2013). In the absence of *Sox3*, the infundibulum does not evaginate fully and cells proliferate less, *Fgf8* and *Bmp4* domains are expanded anteriorly, and RP is bifurcated (Rizzoti *et al*. 2004). This is at least partially a consequence of a slight down-regulation of *Shh* ventrally (Zhao *et al*. 2012) and possibly *Six6*, associated with progenitor proliferation in the eye and pituitary (Li *et al*. 2002). Bifurcations are also observed in *Sox2*^*+/−*^ embryos reflecting redundancy within VD (Kelberman *et al*. 2006). Both murine mutants, *Sox3*^*−/−*^ and *Sox2*^*+/−*^ are affected by mild hypopituitarism and the gland is slightly hypoplastic (Rizzoti *et al*. 2004, Kelberman *et al*. 2006). For SOX3, this is reflecting its role in the hypothalamus where it is maintained, while SOX2 is additionally required in RP (Jayakody *et al*. 2012). Loss of *Sox2* also significantly affects the number of GnRH neurons; therefore, the hypogonadotrophic hypogonadism displayed by human *SOX2* patients is likely to be of hypothalamic origin (Jayakody *et al*. 2012).

In RP, SOX2 is present from at least 9.5 dpc and the protein is maintained in adult pituitary SCs, along with a SOXE sub-family member, SOX9 (Fauquier *et al*. 2008, Andoniadou *et al*. 2013, Rizzoti *et al*. 2013). Deletion of *Sox2* in RP at 12.5 dpc results in reduction of proliferation and, in consequence, endocrine cell deficits where later-born cell types, in particular somatotrophs, are more affected. Expression of the transcription factors PROP1 and PIT1 is downregulated in *Sox2* mutant embryos, but the molecular mechanisms underlying this are not known (Jayakody *et al*. 2012). In conclusion, SOX2 is required within RP for progenitor proliferation.

##### PROP1

PROP1, a paired homoeodomain transcription factor, is the earliest exclusive marker of pituitary identity. In human, mutations are associated with congenital CPHD. In the mouse, PROP1 starts to be expressed at 10 dpc and is then maintained throughout development in SOX2-expressing progenitors except for those in the future IL. Postnatally, it becomes quickly down-regulated and it is present only in a small proportion of SOX2^+^ cells (Gage *et al*. 1996, Sornson *et al*. 1996, Yoshida *et al*. 2009, 2011). Mice homozygous for the *Prop1* null mutant, and the naturally occurring Ames Dwarf mutant, *Prop*^*df/df*^ (which results in low DNA-binding activity), both display strong reduction in PIT1 expression and consequently loss of somatotrophs, lactotrophs, thyrotrophs and also gonadotrophs, while *Hesx1* expression is maintained beyond its normal temporal limit (Gage *et al*. 1996, Sornson *et al*. 1996, Nasonkin *et al*. 2004). As mentioned earlier, PROP1 can interact with β-catenin and this complex activates *Pit1* expression (Olson *et al*. 2006). There must, nevertheless, be another level of regulation for *Pit1* activation as PROP1 is expressed from 10 dpc while *Pit1* is first detected at 13.5 dpc. Moreover, PROP1 probably just initiates *Pit1* expression and is quickly down-regulated, because a maximum of only 9.7% of PIT1-expressing cells also express PROP1 (Yoshida *et al*. 2009). Another aspect of PROP1 function is observed in mutants, where progenitors fail to populate the forming AL, inducing formation of a dysmorphic gland at 14.5 dpc. It is only after birth that, as a consequence of a reduced cell pool in AL, both reduction in proliferation and increased apoptosis result in a hypoplastic gland (Ward *et al*. 2005, 2006). Interaction with NOTCH signalling is proposed to underline the mislocalisation of progenitors (Himes & Raetzman 2009). In summary, PROP1 is initially ubiquitously expressed in progenitors and confers a pituitary identity, while it is required later for morphogenesis of AL.

### Commitment and differentiation of RP progenitors

As RP progenitors exit the cell cycle, they express the negative regulators of cell proliferation p57^KIP^ followed, as they differentiate, by up-regulation of p27^KIP^. Both these proteins prevent cell cycle re-entry (Bilodeau *et al*. 2009). Analysis of mutants, where either cell cycle exits or differentiation is impaired, further reveals that both processes are regulated independently (for review, see Drouin *et al*. (2010)). General control of endocrine differentiation relies at least on the presence of the histone demethylase LSD1, acting both in activator and in repressor complexes (Wang *et al*. 2007), and the zinc finger protein INSM1 (Welcker *et al*. 2013). Deletion phenotypes of either gene are very similar, with a normal pituitary appearance but a block of endocrine differentiation, up-regulation of NOTCH pathway components (Wang *et al*. 2007, Welcker *et al*. 2013) and persistence of SOX2/SOX9 expression (Welcker *et al*. 2013). In the normal pituitary, emergence of each endocrine lineage relies also on the expression of a lineage-specific transcription factor acting as a switch to promote differentiation of a certain lineage while sometimes repressing emergence of others. Molecular events leading to the differentiation of each pituitary endocrine cell type will be described herein.

### Commitment and differentiation of RP progenitors

#### PIT1 lineage: somatotrophs, lactotrophs and thyrotrophs

The POU homoeodomain protein PIT1 is exclusively expressed in the pituitary from 13.5 dpc (Li *et al*. 1990, Simmons *et al*. 1990). Its expression is activated by PROP1 (Olson *et al*. 2006) and maintained in terminally differentiated somatotrophs, lactotrophs and thyrotrophs, where it regulates expression of hormones and hypothalamic peptide receptors. PIT1 is also necessary for *Gh* promoter hypomethylation, associated with active transcription; therefore, it also influences accessibility for other regulators (Massah *et al*. 2014). In *Pit1* mouse mutant embryos, emergence of endocrine cells takes place, but these are not maintained postnatally. Proliferation is reduced and apoptosis occurs, leading to GH, PRL and thyroid-stimulating hormone (TSH) deficiencies. The protein therefore appears to be necessary for postnatal expansion/survival probably in response to both hypothalamic and local signals (Ward *et al*. 2006).

##### Somatotrophs

In the embryo, PIT1 activates the expression of the bHLH factor *Neurod4* at 13.5 dpc. NEUROD4 is required for onset of somatotroph differentiation. In its absence, somatotroph numbers are very low in the embryo, although this improves postnatally. However, these cells never express the receptor for GH-releasing hormone (GHRH, hypothalamic peptide promoting GH secretion), resulting in dwarfism (Zhu *et al*. 2006). The Notch ligand Dlk1 in also expressed by somatotrophs and loss of the gene leads to a mild reduction in GH (Cheung *et al*. 2013). Cross-regulatory mechanisms between different cell types also control endocrine populations: after birth, the histone demethylase LSD1 acts as a co-activator on the *Gh* promoter, while it participates in *Prl* repression (Wang *et al*. 2007).

##### Lactotrophs

The emergence of lactotrophs, mainly postnatally, is thought to largely rely on the concerted transcriptional activities of PIT1 and oestrogen receptors (for review, see Featherstone *et al*. (2012)). It has been initially proposed that lactotrophs could transdifferentiate from somatotrophs; however, cell lineage tracing experiments have shown that this was not a significant phenomenon and that lactotrophs predominantly differentiate from progenitors (Luque *et al*. 2007, Castrique *et al*. 2010, Fu *et al*. 2012).

##### Thyrotrophs

Both thyrotrophs and gonadotrophs express αGSU (the common subunit for TSH and gonadotrophins), the earliest marker of endocrine differentiation, appearing at 11.5 dpc. Therefore, early specification processes, comprising regulators of the *Cga* gene (encoding for αGSU), are shared between the two populations. FOXL2, a forkhead transcription factor, is the first marker of gonadotroph and thyrotroph commitment; expressed ventrally in RP at 10.5 dpc (Treier *et al*. 1998), it persists in these two endocrine cell types until adulthood. LHX3 and LHX4 are required for its expression (Ellsworth *et al*. 2006). FOXL2 can regulate *Cga* expression but does not appear to be essential (Ellsworth *et al*. 2006). *Foxl2*^*−/−*^ pituitaries are hypoplastic; while all endocrine cell types are present, there is an increased cellular density (Justice *et al*. 2011), suggesting a general defective endocrine maturation, probably of hypothalamic origin. Null pituitaries also present more corticotrophs and somatotrophs in males, and reduced *Cga*, *Fsh* (*Fshb*), *Gh* and *Prl* levels in females. This could reflect functions of the protein outside the pituitary; therefore, to better characterise FOXL2 function, the consequences of its conditional deletion in the gonads (see below) and the hypothalamus should be investigated in the pituitary. At 12.5 dpc, the zinc finger transcription factor GATA2, mostly known as an important regulator of haematopoietic SCs, starts to be expressed in the developing pituitary, in the same ventral region as FOXL2. It can also activate expression of *Cga*, and, along with PIT1, that of TSH (Dasen *et al*. 1999). It has been proposed that PIT1 blocks a suppressor region in the TSHβ promoter, allowing access and transactivation by GATA2 (Kashiwabara *et al*. 2009). GATA2 is maintained in thyrotrophs and gonadotrophs (Dasen *et al*. 1999). Conditional deletion of the gene in αGSU-expressing cells causes a reduction in thyrotroph numbers at birth, suggesting that it plays a role in specification and/or expansion of this population. However, this deficiency is transient, and elevation of *Gata3* expression in mutants suggests the existence of a compensatory mechanism (Charles *et al*. 2006). GATA2 is also required later for mature thyrotroph and also gonadotroph function (Charles *et al*. 2006). As mentioned earlier, PITX1 and PITX2 are also present in thyrotrophs, where they can activate *Gata2* expression (Suh *et al*. 2002) and are necessary for endocrine function (Castinetti *et al*. 2011*b*).

#### TPIT lineage: corticotrophs and melanotrophs

The T-box transcription factor TPIT (TBX19) is required for corticotroph and melanotroph differentiation (Pulichino *et al*. 2003*a*,*b*). TPIT expression is first and exclusively observed in RP at 12.5 dpc just before differentiation of the first corticotrophs. Its expression is maintained in mature corticotrophs and melanotrophs. TPIT, along with PITX1 and the ETS factor ETV1, controls *Pomc* expression (Lamolet *et al*. 2001, Lavoie *et al*. 2008, Budry *et al*. 2011*b*). Mutations in both human and murine *TPIT* are associated with severe ACTH deficiencies (Pulichino *et al*. 2003*a*,*b*). Corticotroph commitment is nevertheless observed in murine *Tpit* mutants, but terminal differentiation fails to occur. Moreover, in addition to ‘promoting its own lineage’, TPIT also actively inhibits the emergence of gonadotrophs and rostral-tip thyrotrophs. *In vitro* TPIT and SF1 mutually repress each others' transcriptional activities, by direct protein–protein interaction. The relevance of this interaction is demonstrated *in vivo*, in *Tpit* null IL, by appearance of ectopic gonadotrophs and PIT1-independent thyrotrophs (Pulichino *et al*. 2003*a*,*b*). Finally, network formation is important for optimal POMC expression, because loss of N-cadherin in POMC-expressing cells results in disorganisation of both IL architecture and AL corticotroph network, and a reduction in *Pomc* levels (Himes *et al*. 2011).

##### Corticotrophs

In the context of the pituitary, NeuroD1, a bHLH transcription factor, is transiently expressed only in corticotrophs, where it can also act along with other bHLH proteins and PITX1 to induce the expression of *Pomc* (Lavoie *et al*. 2008). However, corticotroph differentiation is only slightly delayed in its absence (Lamolet *et al*. 2004). *Neurod1* is still expressed in *Tpit* mutants, demonstrating that corticotroph differentiation rather than their commitment is prevented (Pulichino *et al*. 2003*a*,*b*).

##### Melanotrophs

PAX7, a paired box protein, mostly known for its role in muscle satellite cells, has been recently shown to be responsible for melanotroph specification (Budry *et al*. 2012). It is expressed in the future IL from 14.5 dpc, where it briefly co-localises with SOX2, and it is maintained while TPIT is up-regulated in differentiating and mature melanotrophs. Deletion of the gene results in a loss of melanotrophs, which are replaced by ectopic corticotrophs. Melanotroph specification is dependent on the chromatin re-modelling properties of PAX7, which allows TPIT to access a subset of melanotroph-specific enhancers (Budry *et al*. 2012). Finally, proper organisation of IL and its associated dorsal SOX2-expressing progenitor cell layer relies on the presence of the adaptor protein NUMB, probably through its adherens junction-stabilising properties (Moran *et al*. 2011).

#### Gonadotrophs

The first prospective gonadotroph-specific marker is probably the GnRH receptor, expressed from 12.5 dpc, well before gonadotrophins at 16 dpc (Wen *et al*. 2010). Its expression is induced at least in part by LHX3 and ISLET1 (Schang *et al*. 2013). GnRHR is required in the embryo because emergence of follicle-stimulating hormone (FSH)-positive gonadotrophs depends on GnRH (Wen *et al*. 2010). FOXL2 and GATA2, as mentioned earlier, are expressed early and maintained in both thyrotroph and gonadotroph populations (Charles *et al*. 2006, Ellsworth *et al*. 2006). FOXL2 is an important regulator of ovarian development and, in its absence, fertility is impaired (Uhlenhaut *et al*. 2009). Conditional deletion of *Foxl2* in gonadotrophs indicates that the protein is required, along with SMAD4 for *Fsh* expression (Fortin *et al*. 2014). FOXL2 is also likely to be involved in gonadotroph adenoma growth (Chesnokova *et al*. 2012). GATA2 is not essential for gonadotroph development, but FSH levels are reduced in mutants (Charles *et al*. 2006). At 14.5 dpc, the orphan nuclear receptor SF1 starts to be expressed in future gonadotrophs and GATA2 is involved in its activation (Dasen *et al*. 1999). SF1 is expressed and required in the different components of both the reproductive and adrenal hypothalamo–pituitary axis. It can activate expression of *Cga*, *Lh* (*Lhb*), *Fsh* and *Gnrhr* along with co-factors such as early growth response 1 (EGR1) and PITX1 (Fortin *et al*. 2009). Conditional deletion of *Sf1* in αGSU-positive cells results in a dramatic reduction in gonadotrophin expression, but high doses of GnRH can partially rescue this phenotype; therefore, responsive gonadotrophs or precursors are still present (Zhao *et al*. 2001).

## Pituitary SCs

Pituitary SCs had been suggested to exist for a long time, but it is only recently that their existence has been convincingly demonstrated (for reviews, see Rizzoti (2010), Castinetti *et al*. (2011*a*), Davis *et al*. (2011) and Vankelecom (2012)). RP progenitors express SOX2 from early stages, and SOX9 is up-regulated in the SOX2-positive cells towards the end of gestation (14.5 dpc). Its up-regulation correlates with reduced levels of both differentiation and proliferation (Rizzoti *et al*. 2013; C Pires and K Rizzoti, unpublished observations). In the embryonic CNS, SOX9 is required for neural SC generation, (Scott *et al*. 2010). Future investigations may reveal if it has a similar role in the pituitary, operating a switch from embryonic progenitors towards more quiescent SCs. SOX2; SOX9 double-positive cells are maintained postnatally, mainly in an epithelial layer surrounding the pituitary cleft, but some are also scattered in the AL (Fauquier *et al*. 2008). SOX2; SOX9 double-positive cells lining the cleft also express the Glial cell line-derived neurotrophic Factor Receptor GFRα2 (Garcia-Lavandeira *et al*. 2009).

*In vitro*, SOX2- and SOX9-positive cells isolated from adult pituitaries have the capacity to generate spheres (Fauquier *et al*. 2008, Rizzoti *et al*. 2013), a property displayed by progenitor populations in different tissues. Spheres are characterised by self-renewal and differentiation potentials. Pituispheres have a limited self-renewal capacity (for review, see Rizzoti (2010)) and this may reflect sub-optimal conditions, as a transient loss of SOX9 is observed during the early phases of culture (Rizzoti *et al*. 2013). Pituispheres can generate endocrine cells (Fauquier *et al*. 2008, Rizzoti *et al*. 2013), but the molecular mechanisms are unknown. These represent a good model to investigate whether adult progenitors utilise embryonic differentiation processes.

*In vivo*, lineage-tracing experiments using both *Sox2*^*CreERT2*^- and *Sox9*^*CreERT2*^-targeted alleles revealed that cells expressing either (or both) of them can self-renew and give rise to endocrine cells, both in the embryo and postnatally (Andoniadou *et al*. 2013, Rizzoti *et al*. 2013). In the adult, pituitary SCs are mostly quiescent, and they proliferate and differentiate only rarely (Fauquier *et al*. 2008, Andoniadou *et al*. 2013, Rizzoti *et al*. 2013). As mentioned earlier, SOX2 is required for RP progenitor proliferation. In the adult SCs, its role is likely to be different, reflecting interactions with different partners and the effect of niche-derived factors that regulate quiescence vs activation, and self-renewal vs differentiation (for review, see Kamachi & Kondoh (2013)). Additionally, the balance between SOX2 and p27^kip^ is likely to be important in the control of proliferation of pituitary SCs. P27^kip^ is a negative cell cycle regulator but it is also able to recruit co-repressors to down-regulate *Sox2* expression in embryonic SCs (ESCs) and this is important for differentiation to proceed. *In vivo*, *p27*^*kip*^ null mice display intermediate lobe tumours and a thicker SC layer lining the cleft. Deletion of one allele of *Sox2* on this null background rescues these phenotypes, highlighting the physiological relevance of this interaction (Li *et al*. 2012). In RP, p27^kip^ and SOX2 are not expressed in the same cells (Bilodeau *et al*. 2009), but at some point p27^kip^ becomes ubiquitously expressed and it is likely to represent an important regulator of *Sox2* expression.

A role for the NOTCH pathway in proliferation of progenitors had been proposed *in vitro* (Chen *et al*. 2006). Recently, conditional deletion of NOTCH2 in progenitors confirmed this function as numbers are reduced postnatally, and there is also an abnormal localisation of SOX2- and SOX9-expressing cells in mutants (Nantie *et al*. 2014). Co-localisation of SOX2 with the transcription factor PROP1 is observed in AL up until 1 week postnatally, after which expression of the later dramatically decreases (Yoshida *et al*. 2011). This may reflect different rates, or mechanisms, of differentiation. In the adult, there is indeed very little differentiation from SCs under normal conditions (Andoniadou *et al*. 2013, Rizzoti *et al*. 2013). In agreement with this observation, an elegant study, where apoptosis is induced upon cell division, demonstrated that corticotroph turnover relies on proliferation of differentiated cells or self-duplication (Langlais *et al*. 2013). In contrast, physiological challenges such as pituitary target organ ablation efficiently induce proliferation and differentiation of SCs, demonstrating their regenerative potential (Rizzoti *et al*. 2013).

Tumour-forming potential of the SC compartment has been recently examined postnatally by expressing a degradation-resistant form of β-catenin that was conditionally expressed under the control of *Sox2*^*CreERT2*^ and tamoxifen administration. Tumours are formed, but surprisingly they were not composed of mutant SCs. Instead, the SCs initially form clusters that subsequently induce neighbouring cells to form the tumours in a paracrine manner (Andoniadou *et al*. 2013).

In conclusion, pituitary SCs do not significantly participate in adult cell turnover but they have a regenerative potential. They have a tumourigenic potential as they can induce tumours if mutated (Andoniadou *et al*. 2013), but they have not yet been shown to form tumours themselves.

## *In vitro* recapitulation of pituitary ontogeny

*In vitro* production of endocrine cells has proved to be difficult and inefficient until recently when two strategies were devised that successfully reproduced some of the embryonic events involved in pituitary development as described earlier, allowing endocrine cells to be obtained from ESCs (Suga *et al*. 2011, Dincer *et al*. 2013; Fig. 3). In the late Yoshiki Sasai's laboratory, Wataya *et al*. (2008) had previously been able to induce hypothalamic identity in 3D mouse ESC aggregates. By further inducing rostral character, they reasoned that it might be possible to obtain ANR-like territory apposed to neuroectoderm-like tissue, where RP may develop. By treating large aggregates with BMPs, which at the placodal stage induce ectodermal identity (for review, see Saint-Jeannet & Moody (2014)), they could induce expression of PITX1 and PITX2 in a superficial layer surrounding a RAX-positive neurectodermal domain. Superposition of these two territories was shown to be essential, and also sufficient for further pituitary-like development, mimicking events *in vivo*. Subsequent exposure to HH agonist was sufficient to induce LHX3 expression in the PITX2^+^ layer, initially in cell clusters that thickened, and then invaginated to form spectacular RP-like structures. Inhibition of NOTCH signalling resulted, as again reported *in vivo* (Zhu *et al*. 2006, Kita *et al*. 2007), in differentiation of corticotrophs in these pouches. Their functionality was demonstrated after transplantation *in vivo* in hypophysectomised mice. Obtention of other endocrine cell types was less efficient, perhaps because the absence of vascularisation compromises endocrine differentiation and maturation, as observed in organoids (for review, see Lancaster & Knoblich (2014)). Activation of Wnt signalling induced PIT1 expression, which could reflect cooperation of β-catenin with PROP1 (Olson *et al*. 2006). Somatotrophs and lactotrophs were further differentiated using, respectively, glucocorticoids and oestradiol, both supplemented with insulin (Suga *et al*. 2011). Using human ESCs, Dincer and collaborators, in Studer's laboratory, used a different approach and were able after complex sequential modulation of different pathways to directly induce a placodal fate. Importantly, they succeeded in adherent cultures (Dincer *et al*. 2013). Briefly, dual SMAD inhibition was initially performed to impart neural fate, and the subsequent de-repression in combination with FGF inhibition was sufficient for acquisition of placodal identity. Modulation of FGF, BMP and SHH pathways further allowed specification of lens, trigeminal and pituitary placode identity. As reported by Suga *et al*. (2011) treatment with HH agonist resulted initially in HP character (PITX1; SIX6^+^) and further RP identity (LHX3^+^). But in contrast with Suga *et al*. (2011) ACTH expression was then observed without further treatment, while induction of *PIT1* and *GATA2* expression relied on NOTCH pathway inhibition. *In vivo* secretion was demonstrated after subcutaneous implantation in mice (Dincer *et al*. 2013). In both studies, ACTH-positive cells were by far the most efficiently generated cell type. In the future, implantation of cells in the pituitary should be evaluated as hormone secretions are normally controlled locally by the hypothalamus. It will also be necessary to assess the efficiency of these protocols with induced pluripotent SCs.

## Conclusions

Significant advances have been made in recent years and we understand better as to how RP progenitors are controlled and how endocrine cells differentiate, and, importantly, we know that they form endocrine networks. The generation of endocrine cells from ESCs and their subsequent transplantation *in vivo* represent exciting progress towards the use of regenerative medicine to treat endocrine deficits or manipulate endocrine outputs. We still need a better understanding of how cell fates are specified *in vivo*, as embryonic progenitors exit the cell cycle, for efficient *in vitro* generation of all endocrine cell types. In addition, the recent characterisation of pituitary SCs opens the alternative possibility of direct somatic cell conversion into organ-specific SCs for use in regenerative medicine.

## Figures and Tables

**Figure 1:** Development and function of the pituitary–hypothalamic axis. Pituitary development is initiated with the appearance of the hypophyseal placode, apposed to the future ventral diencephalon. The placode later invaginates to become Rathke's pouch (RP), still in contact in its dorsal most part with the infundibulum, which lies within the ventral diencephalon. The infundibulum then evaginates towards RP. It will give rise to the median eminence, the pituitary stalk and the posterior lobe, while the anterior and intermediate lobes originate from RP. Postnatally, the hypothalamus centralises peripheral information and controls pituitary endocrine secretions through release of hypophysiotrophic hormones. Hypothalamic peptide hormones can reach the gland directly, such as oxytocin and vasopressin secreted directly in the posterior lobe, or via the hypophyseal portal system; peptides (GnRH, gonadotrophin-releasing hormone; GHRH, GH-releasing hormone; TRH, thyrotropin-releasing hormone; CRH, corticotropin-releasing hormone; and the inhibitory SST, somatostatin) are secreted at the median eminence and collected by capillaries (adapted from Rizzoti & Lovell-Badge (2011)). Anterior pituitary endocrine cells comprise lactotrophs (producing prolactin, Prl), gonadotrophs (producing luteinizing hormone, LH; and follicle stimulating hormone, FSH), thyrotrophs (producing thyroid stimulating hormone, TSH), corticotrophs (producing adrenocorticotrophic hormone, ACTH; proteolytically cleaved from proopiomelanocortin, POMC) and somatotrophs (producing growth hormone, GH).

**Figure 2:** Main signalling pathways and factors required during pituitary development. Opposing activities of BMP4 and SHH within the ventral diencephalon pattern this region and participate in correct morphogenesis of the infundibulum and in consequence positioning of RP. Within the infundibulum, BMP4 and FGF8, FGF10 and FGF18 are required for development of RP. In RP at 10.5 dpc, BMP2 is present and there is a uniform SMAD activation profile, while the FGF pathway is only activated dorsally (Davis *et al*. 2011). At this stage, different transcription factors required for RP progenitor proliferation and/or maintenance are ubiquitously expressed. Later, at 14.5 dpc, progenitors are confined around the RP lumen, while differentiating and differentiated cells away from the lumen define the developing anterior pituitary.

**Figure 3:** *In vivo* and *in vitro* regenerative potential of stem cells in the pituitary. *In vivo*, pituitary SCs can be stimulated by physiological challenge, proliferate and differentiate into the appropriate endocrine cell type. *In vitro*, different strategies have been successfully devised to obtain transplantable endocrine cells. Using mouse ES cells, Suga *et al*. (2011) were able to recapitulate early pituitary development and mimic RP morphogenesis in 3D aggregates (Suga *et al*. 2011). Endocrine cells were further differentiated. Transplantation in hypophysectomised mice demonstrated that these cells were functional. Dincer *et al*. (2013) were also able to differentiate endocrine cells from human ES cells, in adherent cultures, initially by inducing placodal fate, then hypophyseal identity. Transplantation demonstrated *in vivo* secretion. These are significant steps towards regenerative medicine to cure long-term pituitary endocrine deficiencies.
